The article "Martial Arts Competitive Decision-Making Algorithm Based on Improved BP Neural Network" was retracted in 2023. Reasons: unreliable results or conclusions; concerns about the data; concerns about the peer review; concerns about the citations.

# Martial Arts Competitive Decision-Making Algorithm Based on Improved BP Neural Network

**DOI:** 10.1155/2021/9920186

**Published:** 2021-05-11

**Authors:** Huipeng Lv

**Affiliations:** Northeast Petroleum University, Daqing, Heilongjiang, 63318, China

## Abstract

The main body of modern Chinese martial arts competition is the strategy, and fighting has just started in sports competitions. Strategy and action correspond to each other and practice as a set. Therefore, constructing the Chinese martial arts competition decision-making algorithm and perfecting the martial arts competition are intuitive and essential. The formulation of martial arts competition strategies requires scientific analysis of athletic data and more accurate predictions. Based on this observation, this paper combines the popular neural network technology to propose a novel additional momentum-elastic gradient descent. The BP neural network adapts to the learning rate. The algorithm is improved for the traditional BP neural network, such as selecting learning step length, the difficulty of determining the size, and direction of the weight, and the learning rate is not easy to control. The experimental results show that this paper's algorithm has improved both network scale and running time and can predict martial arts competition routines and formulate scientific strategies.

## 1. Introduction

From the concept of martial arts [1, 2], martial art is a traditional sport with Chinese culture as the theoretical foundation, martial arts methods as the primary content, and routines, fighting, and exercises as the primary forms of sports. The types of martial arts mainly include routines, fighting, actions, and exercises. In the context of the current globalization of competitive ideas, competitive sports are the general trend, so the routines or fighting we talk about refer to competitive events. The routines have taken shape, and only Sanda has become a formal event for fighting. Gongfu is the essential skill of martial arts practice [3]. Both routines and fighting must be practiced. Here, we focus on fighting. From the essential core of martial arts, the athletes should be focused on fighting. For example, routines' formation is to preserve some practical fighting techniques and movements in routines and follow fixed rules and sequence arrangement, thus forming a routine. Some movements in the routine can also clearly see the traces of fighting [4]. When explaining routine movements, imaginary movements will hit the opponent's neck, eyes, ribs, crotch, and other parts to make the opponent lose combat effectiveness, preserving the purpose of killing the other party.

From Figure 1, we can see that the content of the routine is quite rich, but the content of the fighting is relatively barren. Therefore, this paper believes that the Chinese martial arts competitive fighting system is not perfect, and the Chinese martial arts competitive fighting project has yet to be developed. From the comparison with the routine, it can be seen that Sanda in fighting includes kicking, hitting, and throwing in martial arts, which can be compared with all kinds of boxing in the routine [5]. The form of movement of pushing hands should be regarded as the transition from the gong method to fighting, which is the mastery of both parties' strength. In the comparison test, the short soldier is also skinny in the four types of equipment in the comparison routine: long, short, double, and soft. Besides, strategic martial art is still the primary manifestation of martial arts.

The article "Martial Arts Competitive Decision-Making Algorithm Based on Improved BP Neural Network" was retracted in 2023. Reasons: unreliable results or conclusions; concerns about the data; concerns about the peer review; concerns about the citations.

However, the strategies of strategic martial arts are ever-changing, with various forms and styles [6]. The formulation of scientific and reasonable martial arts competition strategies can improve the level of competition. The rapid development of neural networks [7–9] and deep learning [10, 11] provides us with new ideas for formulating martial arts strategies. Because artificial neural networks do not need to determine the mapping relationship's mathematical equations between input and output in advance, they can learn specific rules only through training [12]. Set the input value to get the result closest to the expected output value. An artificial neural network's core to realize its function is the algorithm as an intelligent information processing system. BP neural network is a multilayer feed-forward network trained by error backpropagation [13, 14].

This paper combines the popular neural network technology to propose a novel additional momentum-elastic gradient descent based on the above observations. The BP neural network adapts to the learning rate. The algorithm is improved for the traditional BP neural network, such as selecting learning step length, the difficulty of determining the size and direction of the weight, and the learning rate is not easy to control. The experimental results show that this paper's algorithm has improved both network scale and running time and can predict martial arts competition routines and formulate scientific strategies.

The following are the main contributions points of this paper:

1. A novel additional momentum-elastic gradient descent-adaptive learning rate BP neural network is proposed. This algorithm is aimed at the traditional BP neural network, which is difficult to determine the learning step size, weight size, and direction, and the learning rate is not easy to control. And other issues were improved.
2. This paper preliminarily constructs a martial arts competitive strategy algorithm, introduces a neural network algorithm for martial arts strategy, and references related parts of competitive sports.
3. We also constructed a dataset and conducted experiments. The experimental results show that the method in this paper is superior to some current advanced methods.

The article "Martial Arts Competitive Decision-Making Algorithm Based on Improved BP Neural Network" was retracted in 2023. Reasons: unreliable results or conclusions; concerns about the data; concerns about the peer review; concerns about the citations.

The rest of the paper is organized as follows. In Section 2, a background study is given, followed by the methodology in Section 3. In Section 4, experimental setup and result discussion are presented, followed by a conclusion in Section 5.

## 2. Background

The concept of martial arts is defined in “Cihai” Martial arts, also known as “Wuyi” and “National Martial Arts.” Traditional Chinese sports are based on offensive and defensive combat actions such as kicking, beating, falling, holding, falling, smashing, hitting, and stabbing. It is composed of a particular movement pattern. It is divided into two forms: routine and confrontation. The former is divided into boxing and equipment; the latter can be divided into Sanshou, push hands, long soldiers, short soldiers, and so on [15]. According to the characteristics of sports and technical forms, there is internal and external Home, divided into long boxing and short boxing. The definition of sports is explained in Cihai: physical exercise [16] is the primary method, combined with natural factors such as sunlight, air, water, and hygiene measures and organized and planned exercise of the body and mind A type of social activity. Its purpose is to strengthen physical fitness, improve sports skills, enrich cultural life, and cultivate moral sentiment. It is an integral part of social and cultural education. At that time, martial arts were fighting skills to kill opponents and protect themselves. Since New China's founding, martial arts' combative nature has been replaced by modern sports [17, 18], and martial arts have been defined as a sport. Competitiveness refers to competition in sports. “Competition refers to competition and competition,” and skill refers to sports skills. “Competitive sports have the characteristics of competition,” standardization, fairness, clustering, openness, and appreciation.

Chinese martial arts [19] have a long history. Generally, martial arts' historical development is divided into three stages: ancient, modern, and modern. The essence of Chinese ancient martial arts is fighting, so martial arts' historical development is the historical development of fighting. Wushu routines came into being after fighting, and the creation of routines is also for better fighting. Until modern competitive martial arts used “high, difficult, beautiful, new” as the criterion, it was divided into two types of martial arts, routines and fighting Confucian founder Confucius emphasized that both civil and martial arts should be “benevolent in terms of the theoretical awareness of martial arts” [20]. One of the core content of martial arts. Mo Di, the Mo School founder, advocated universal love and nonaggression, supported force, and used force to resist all aggression and injustice. He became the representative and birthplace of “chivalrous” in later generations and a typical chivalrous spirit in history. Some thoughts of the Taoist school have a significant influence on martial arts thought, especially the Taoist understanding of the origin of the universe, such as the understanding of Tao and Qi, the unity of nature and man, and the theory of rigidity and softness, which established the theory and philosophy of martial arts. There are also many places where martial arts absorb the doctrine of military strategists. For example, false moves and feint attacks are drawn from “soldiers are not tired of deceit,” and the understanding of tactics and the grasp of timing are all borrowed from strategists. Including the five elements of yin and yang theory developed from the Book of Changes at that time, it has contributed a lot to the establishment of Tai Chi, Xingyiquan, Baguazhang, and other types of boxing. These simple dialectics have enriched the theory of martial arts and led martial arts to a broad road.

The article "Martial Arts Competitive Decision-Making Algorithm Based on Improved BP Neural Network" was retracted in 2023. Reasons: unreliable results or conclusions; concerns about the data; concerns about the peer review; concerns about the citations.

The artificial neural network is a nonlinear processing system with the input layer, hidden layer, and output layer formed by many processing units interconnected. The artificial neural network is a mathematical model inspired by humans' or animals' neural network functions to process information. This mathematical model's application is similar to the recognition, memory, data analysis, and information processing of the human brain [21]. In processing information, the input layer has different input quantities *x*, and each input quantity *x* has an associated weight *w* corresponding to it. The input volume enters the neural network from the input layer, passes through the stimulation of the weight threshold and the weighted summation, and obtains the output *y*. The output results from the layer under the activation function's perception and continues the following layer's role. In this way, until input quantity is output from the output layer, the error between the output value and the expected value is the smallest. That is, it has three essential elements: connection weight, summation unit, and activation function. The processing unit model is shown in Figure 2.

The article "Martial Arts Competitive Decision-Making Algorithm Based on Improved BP Neural Network" was retracted in 2023. Reasons: unreliable results or conclusions; concerns about the data; concerns about the peer review; concerns about the citations.

There are quite a lot of classification standards for artificial neural networks. ANN can be classified into feed-forward networks and feedback networks based solely on the network structure. Feed-forward neural networks include single-layer and multilayer feed-forward networks. Throughout the ANN application field, feed-forward neural networks are the most frequent and can successfully achieve the expected results. The feed-forward neural network's latest output is not related to the previous output state and is only determined by the current excitation function and weight matrix [22]. Compared with the feed-forward neural network, the feedback neural network is complex and advanced. Its latest output is closely related to the previous output and the latest input, and its intelligence is evident with the associative memory function. It is worthy of promotion and application under the guidance of artificial intelligence. The most commonly used and classic feed-forward neural network is the error backpropagation neural network, referred to as BP neural network.

## 3. Methodology

In this section, the methodology is discussed in detail.

### 3.1. BP Neural Network

BP neural network, the error backpropagation neural network, is the most widely used artificial neural network model. It was proposed by Kůrková in 1985 and gave practical guidance in solving the learning and training problems of multilayer neural networks and gave a comprehensive analysis and derivation in mathematics [21]. The BP neural network's network structure is simple and mainly has three layers: the input layer, hidden layer, and output layer, as shown in Figure 3.

The three-layer BP neural network is shown in Figure 3. In this figure, the number of input nodes is *M*, the number of output nodes is *L*, the initial number of hidden layers is *u*, and the BP neural network's actual input is *x*_1_, *x*_2_,…, *x*_*M*_. The actual output is *y*_1_, *y*_2_,…, *y*_*L*_, the target output is *T*_*k*_, and the output error is *e*_*k*_. Secondly, the input layer's connection weight to the hidden layer is *w*_*ij*_ that the weight can also be called a weight vector. The connection weight from the hidden layer to the output layer is the size and direction of these two weights may be different. The improved BP neural network can modify it to make it develop toward the desired size.

The BP neural network is vividly understood as a supervised learning relationship between teachers and students. It consists of the forward propagation of the first stage signal and the backpropagation of the second stage error [22]. In the first forward propagation, the given signal first enters the network from the input layer and then is pushed by the hidden layer to the output layer. Finally, the signal is transmitted by the output layer. The first stage is completed. The weight of the network is maintained during the entire transmission of the early stage. Consistently, the neurons' state in the next layer is only constrained by the previous layer's neurons. Suppose the result of the signal transmitted from the output layer is far from the expected result. In that case, it will immediately go to the second stage of the error backpropagation learning process. This process is a process of reducing the error. The actual output value is different from the expected value. The difference is used as a new signal input from the output layer, layer by layer, backpropagation to the first input layer, and continue. Continue until the final actual output is closer to the expected value; that is, the error is minimized. In the process of backpropagation, the weight is mainly modified to obtain the desired result. Among them, the changes of other factors also play a supporting role.

The article "Martial Arts Competitive Decision-Making Algorithm Based on Improved BP Neural Network" was retracted in 2023. Reasons: unreliable results or conclusions; concerns about the data; concerns about the peer review; concerns about the citations.

### 3.2. Improved BP Neural Network

Aiming at the shortcomings and limitations of the steepest descent BP neural network and the momentum BP neural network, a new algorithm is proposed: additional momentum-elastic gradient descent-adaptive learning rate BP neural network. First, the learning step's selection and the weight size and direction have been improved, and the learning rate and momentum terms have been limited. Then, the improved new algorithm and the first two BP neural networks are compared and analyzed by simulation experiments, and the correctness, error, and prediction time are calculated. Other indicators found that the new algorithm has higher accuracy, minor errors, fewer iterations, and better overall performance. Finally, the improved BP neural network used in the next chapter of this paper has laid a strong foundation for predicting martial arts strategies.

#### 3.2.1. SDBP Neural Network

The SDBP neural network's learning process [23] is also composed of two stages: the forward propagation of the first stage signal and the second stage error's backpropagation. The weight *w*_*ij*_ and the threshold *a*_*j*_ from the input layer to the hidden layer are continuously adjusted. The weight *w*_*jk*_ from the hidden layer to the output layer and the threshold *b*_*k*_ are modified until the output result is almost the same as the expected result. The SDBP neural network structure is shown in Figure 4, assuming the number of nodes in the input layer, hidden layer, and output layer. They are *M*, *u*, and *L*. The calculation formulas for each layer are as follows.

The article "Martial Arts Competitive Decision-Making Algorithm Based on Improved BP Neural Network" was retracted in 2023. Reasons: unreliable results or conclusions; concerns about the data; concerns about the peer review; concerns about the citations.

Let *k* be the number of iterations; the calculation formula for weight update is

(1) $$\begin{array}{c} w_{k+1}=w_{k}-\alpha g_{k}. \end{array}$$

The weight of the kt iteration *α* is the learning rate, which can be set reasonably during training. The initial default learning rate is 0.01.

Average method: take the average of the three channels' pixels in the RGB image as the gray value of the gray image.

(2) $$\begin{array}{c} g_{k}=\frac{\partial E_{k}}{\partial w_{k}}, \end{array}$$

where *g*_*k*_ is the gradient vector of the *k* th iteration, *E*_*k*_ is the total error performance function of the neural network output of the *k* th iteration, and the output formula of the hidden layer is

(3) $$\begin{array}{c} H_{j}=\sum_{i=1}^{n}w_{ij}x_{i}+a_{j}. \end{array}$$

The input vector *H*_*j*_ is the hidden layer's actual output, *a*_*j*_ is the threshold from the input layer to the hidden layer, and *w*_*ij*_ is the weight from the input layer to the hidden layer. The output formula of the output layer is as follows:

(4) $$\begin{array}{c} O_{k}=\sum_{j=1}^{l}H_{j}w_{jk}+b_{k}. \end{array}$$

The output layer's actual output *b*_*k*_ is the threshold from the hidden layer to the output layer and *w*_*jk*_ is the weight from the hidden layer to the output layer. The calculation formula is as follows:

(5) $$\begin{array}{c} E_{k}=\frac{1}{2}{\sum_{i=1}^{k}\left(Y_{i}-O_{i}\right)}^{2}, \end{array}$$

where *E*_*k*_ is the total error performance function of the neural network output of the *k* th iteration, *Y*_*i*_ is the expected value of the *i* th iteration, and *O*_*i*_ is the actual output of the *i* th iteration.

From equations 1–5 and each layer's function, the surface gradient *g*_*k*_ of the total error of the *k* th iteration can be obtained, and equation 1 is, respectively, introduced. The weight of each layer is revised to ensure that the absolute error is reduced. The small development direction is reduced to the minimum, thus in line with the expected error.

It can be seen from Figure 5 that there are too many minimum points on the error surface because the transfer function of the SDBP neural network is nonlinear.

#### 3.2.2. MOBP Neural Network

MOBP neural network introduces momentum factor *η*(0 < *η* < 1) based on SDBP neural network:

(6) $$\begin{array}{c} \Delta w_{k+1}=\eta \Delta w_{k}+\alpha \left(1-\eta \right)\frac{\partial E_{k}}{\partial w_{k}}, \end{array}$$

where *η* is the momentum factor, *w*_*k*_ is the weight of the *k* th iteration, Δ*w*_*k*_ is the weight correction of the *k* th iteration, *α* is the learning rate, and *E*_*k*_ is the total error performance function.

The article "Martial Arts Competitive Decision-Making Algorithm Based on Improved BP Neural Network" was retracted in 2023. Reasons: unreliable results or conclusions; concerns about the data; concerns about the peer review; concerns about the citations.

The new correction amount of the algorithm is closely related to the previous correction result and restricted. Suppose the last amount correction is too significant. In that case, the sign of the second term of equation 6 is the opposite of the previous correction amount, resulting in the current correction. If the last revision is too minor, the second term of equation 6 is the same as the previous correction sign. As a result, the correction is increased, and the training speed will be improved for the network. Therefore, the MOBP neural network essentially increases the correction in the same gradient direction, that is, increases the “momentum” in the same gradient direction by increasing the momentum factor *η* reasonably.

In the MOBP neural network, compared to the SDBP neural network's learning rate, the MOBP neural network's learning rate can be increased to a greater extent. Still, the increased learning rate will not make the network training impossible and paralyzed. There are two reasons. On the one hand, when the degree of correction is too large, the algorithm can correct to decrease, ensuring that the correction direction still maintains the direction of convergence. On the other hand, MOBP neural network does the same by introducing momentum factor. The correction amount of the gradient direction is reasonably increased to increase the learning rate. From this, it can be obtained that, based on ensuring the algorithm's stability, the MOBP neural network's learning time is shortened, and the convergence speed has been dramatically improved.

#### 3.2.3. Limitations of BP Neural Network

When applying artificial neural network modeling in related fields, most neural network models use BP neural network, SDBP neural network, MOBP neural network, and other improved forms. However, BP neural network still has its limitations.

1. The limitations of the network itself: the BP neural network is a static transmission network. It can only complete nonlinear static mapping safely and does not have the information processing function that changes dynamically with time or space.
2. Selection of initial parameters: It is difficult for BP neural network to select initial parameters, especially the size and direction of initial weights and thresholds. Although there are correction formulas, once the initial values are determined, it is equivalent to determining the network convergence. When network learning is over, it will generally converge to the local extreme value closest to the initial value, directly affecting the difference between the local extreme point's error and the ideal error.
3. The choice of learning step length: The training step length in BP neural network is a fixed value, and the path left by the gradient method is zigzag when approaching the minimum point. The closer to the minimum point, the faster the convergence speed. Therefore, to reduce the error, the training step length should be set as small as possible. If the step length is too small, the training time will increase, which leads to the difficulty of establishing the training step length. To obtain relevant learning results, it generally needs to be rich practical experience or repeated adjustments to the step length.
4. The choice of learning rate: If the learning rate is selected too large, it will make learning unstable; on the contrary, if the learning rate is chosen too small, it may increase the learning time and cause network paralysis. At present, a fast and reasonable method has not been explored, to solve the difficulty of selecting the learning rate of BP neural network.

The article "Martial Arts Competitive Decision-Making Algorithm Based on Improved BP Neural Network" was retracted in 2023. Reasons: unreliable results or conclusions; concerns about the data; concerns about the peer review; concerns about the citations.

### 3.3. Improved BP Neural Network

Because of the limitations of the SDBP neural network, that is, MOBP neural network and BP neural network, this paper first improves the selection of learning step size and the size and direction of weights then enhances the selection of learning rate, that is, the new algorithm, that is, BP neural network with additional momentum-elastic gradient descent-adaptive learning rate.

The selection of the learning step length in the BP neural network is essential. If the step length is too large, the network will converge quickly, but it will cause instability in network learning; too small a step length can avoid instability, but the convergence speed will slow down. Solving this contradiction, it is proposed to add an “additional momentum term,” based on SDBP neural network and MOBP neural network, add a correction value proportional to the previous weight or threshold value in the correction of each layer weight or threshold, and recalculate the new weight (or threshold) correction amount according to the backpropagation method. The specific adjustment formula is as follows:

(7) $$\begin{array}{c} \Delta w_{ij}\left(n\right)=\lambda \Delta w_{ij}\left(n-1\right)+\zeta \delta_{j}\left(t\right)v_{i}\left(n\right), \end{array}$$

(8) $$\begin{array}{c} \Delta b_{i}\left(n\right)=\lambda \Delta b_{i}\left(n-1\right)+\zeta \delta_{i}\left(t\right), \end{array}$$

where *n* is the number of trainings, *λ* is the momentum term, *ζ* is the learning step size, Δ*w*_*ij*_(*n*) is the correction of the weight of the *n* th training, Δ*b*_*i*_(*n*) is the correction of the *n* th training threshold, and *δ*_*j*_(*t*)*v*_*i*_(*n*) is the *n* th training gradient vector. Write equation 8 as a time series *t* as a variable *t* ∈ [0, *n*]; then, equation 8 can be regarded as the first-order difference equation Δ*w*_*ij*_(*n*). The calculation equation is as follows:

(9) $$\begin{array}{c} \Delta w_{ij}\left(n\right)=\zeta \sum_{t=0}^{n}\lambda^{n-1}\delta_{j}\left(t\right)v_{i}\left(n\right),\\ \delta_{j}\left(t\right)v_{i}\left(n\right)=-\frac{\partial E\left(n\right)}{\partial w_{ij}\left(n\right)}, \end{array}$$

where *δ*_*j*_(*t*)*v*_*i*_(*n*) is understood as the gradient vector of the *n* th training; then

(10) $$\begin{array}{c} \Delta w_{ij}\left(n\right)=-\zeta \sum_{t=0}^{n}\lambda^{n-t}\frac{\partial E\left(n\right)}{\partial w_{ij}\left(n\right)}. \end{array}$$

In the training process of the additional momentum method, to prevent the corrected weight from having an excessive influence on the error, the momentum term *λ* needs to be strengthened; that is, the judgment condition of the additional momentum method in the training process is

(11) $$\begin{array}{c} \lambda =\left\{\begin{array}{cc} 0, & E\left(n\right)>1.04E\left(n-1\right),\\ 0.95, & E\left(n\right)<E\left(n-1\right),\\ \lambda , & \text{otherwise.} \end{array}\right. \end{array}$$

However, the additional momentum BP neural network algorithm's hidden layer generally uses an S-type activation function. The S-type function is often called a “squeeze” function because it can compress an infinite input range to a limited output range. When the input is significant, the slope is almost close. It will cause the gradient amplitude in the algorithm to be tiny, making the correction process meaningless. In response to this problem, the elastic gradient descent method is introduced to improve again. The elastic gradient descent method does not study the amplitude of the partial derivative. Only the partial derivative sign is studied to determine the weight's update direction, and the revised “update value determines the size of the weight change.” If the sign of the partial derivative of the objective function to a certain weight is in two consecutive iterations and if the medium is unchanged, increase the corresponding “update value”; otherwise, decrease the corresponding “update value.” Use the additional momentum method and the elastic gradient descent method to improve the BP neural network at the same time. It will provide the range, the size of the correction, the number of weights, and the direction of updating the weights. It can also significantly prevent the training process from falling into a local minimum and speed up the convergence speed.

The article "Martial Arts Competitive Decision-Making Algorithm Based on Improved BP Neural Network" was retracted in 2023. Reasons: unreliable results or conclusions; concerns about the data; concerns about the peer review; concerns about the citations.

## 4. Experiments

### 4.1. Experimental Environment

Since the experiment in this paper needs to train a deep neural network, the scale is large, the structure is more complex, and the calculation scale is enormous. The programming language used is Python, the version is 3.6, the deep learning framework used is Keras 2.1.5, and the IDE for program deployment is Pycharm. All experiments are conducted in the same environment. All our experiments have been conducted on a desktop PC with an Intel Core i7-8700 processor and an NVIDIA GeForce GTX 1080ti GPU.

### 4.2. Datasets Preprocessing

The data set used in this paper is collected in martial arts competitions. This paper removes singular values and unstable values and creates training sets and test sets.

### 4.3. Experimental Results

All experiments are performed on the same platform, and the experimental results are expressed in terms of error rate and prediction time. The experimental results comparing various algorithms are shown in Table 1 below.

It can be seen from Table 1 that the MDBP neural network adds a momentum term based on the SDBP neural network to modify the weight and threshold. Its test error rate is lower than that of the DBP neural network. About 2 percentage points reduce the error rate. The new algorithm in this paper has improved the selection of learning step size and the size and direction of weights and limited the choice of momentum and learning rate, making the new algorithm more efficient. The error rate is significantly lower than that of other algorithms, and nearly 5 percentage points significantly reduce the new algorithm. From the comparison of error rates in Table 1, it can be fully seen that the error rate of the new BP neural network is significantly lower than the other two BP neural network lines and has a better prediction effect.

It can be seen from Table 2 that the improvement of the MOBP neural network over the SDBP neural network is the introduction of a momentum term; that is, a more significant learning rate can be used without paralyzing the learning process. The MOBP neural network always accelerates the same gradient direction. The correction amount, that is, the MABP neural network, has a faster convergence rate than the SDBP neural network, and the learning time is shorter. The new algorithm is more aimed at the selection of the first learning step. The size and direction of the weights are improved, and the momentum term is improved. There are clear criteria for selecting learning rate; that is, the new algorithm can fine-tune the correction of weights and increase the learning rate within a reasonable range and at the same time accelerate the convergence speed, that is, reduce the prediction time. The comparison can clearly show that the new algorithm's prediction time is significantly lower than that of the other two types of algorithms through the prediction time.

The article "Martial Arts Competitive Decision-Making Algorithm Based on Improved BP Neural Network" was retracted in 2023. Reasons: unreliable results or conclusions; concerns about the data; concerns about the peer review; concerns about the citations.

## 5. Conclusion

The formulation of martial arts competitive strategies requires scientific analysis of competitive data and more accurate predictions. Based on this observation, this paper combines the popular neural network technology. It proposes a novel additional momentum-elastic gradient descent-adaptive learning rate BP neural network. The algorithm is improved for the traditional BP neural network, such as selecting learning step size and the difficulty of determining the weight's size and direction. The learning rate is not easy to control. The experimental results show that this paper's algorithm has made good improvements in both in-network scale and running time and can predict martial arts competition routines and formulate scientific strategies.

## Figures and Tables

**Figure 1:** The schematic diagram of martial arts content classification.

**Figure 2:** Artificial neural network model diagram.

**Figure 3:** The structure of BP neural network.

**Figure 4:** The structure of SDBP neural network.

**Figure 5:** Error surface plot.

**Table 1:** Test error rate of different types of martial arts BP neural network (%).

Type	SDBP	MOBP	Ours
Optional boxing	6.23	4.85	1.37
Prescribed boxing	7.35	5.97	1.78
Traditional boxing	7.69	6.23	2.03
Short instrument	8.23	5.14	1.99
Long instrument	6.58	4.69	1.87
Double instrument	7.69	5.28	2.01
Soft instrument	8.59	4.99	1.89

**Table 2:** The prediction time of BP neural network for different martial arts(s).

Type	SDBP	MOBP	Ours
Optional boxing	37.3	23.6	17.2
Prescribed boxing	34.5	24.5	18.3
Traditional boxing	35.9	22.9	15.2
Short instrument	36.5	23.8	16.3
Long instrument	35.9	24.9	15.2
Double instrument	37.5	25.8	17.2
Soft instrument	35.9	24.9	18.3

## Data Availability

The data used to support the findings of this study are included within the article.
